# Deep Learning-Based Multimodal 3 T MRI for the Diagnosis of Knee Osteoarthritis

**DOI:** 10.1155/2022/7643487

**Published:** 2022-04-29

**Authors:** Yong Hu, Jie Tang, Shenghao Zhao, Ye Li

**Affiliations:** Department of Orthopaedic, Wuhan Fourth Hospital, Wuhan, 430000 Hubei, China

## Abstract

The objective of this study was to investigate the application effect of deep learning model combined with different magnetic resonance imaging (MRI) sequences in the evaluation of cartilage injury of knee osteoarthritis (KOA). Specifically, an image superresolution algorithm based on an improved multiscale wide residual network model was proposed and compared with the single-shot multibox detector (SSD) algorithm, superresolution convolutional neural network (SRCNN) algorithm, and enhanced deep superresolution (EDSR) algorithm. Meanwhile, 104 patients with KOA diagnosed with cartilage injury were selected as the research subjects and underwent MRI scans, and the diagnostic performance of different MRI sequences was analyzed using arthroscopic results as the gold standard. It was found that the image reconstructed by the model in this study was clear enough, with minimum noise and artifacts, and the overall quality was better than that processed by other algorithms. Arthroscopic analysis found that grade I and grade II lesions concentrated on patella (26) and femoral trochlear (15). In addition to involving the patella and femoral trochlea, grade III and grade IV lesions gradually developed into the medial and lateral articular cartilage. The 3D-DS-WE sequence was found to be the best sequence for diagnosing KOA injury, with high diagnostic accuracy of over 95% in grade IV lesions. The consistency test showed that the 3D-DESS-WE sequence and T2∗ mapping sequence had a strong consistency with the results of arthroscopy, and the Kappa consistency test values were 0.748 and 0.682, respectively. In conclusion, MRI based on deep learning could clearly show the cartilage lesions of KOA. Of different MRI sequences, 3D-DS-WE sequence and T2∗ mapping sequence showed the best diagnosis results for different degrees of KOA injury.

## 1. Introduction

Knee joint is the largest and most complicated joint in human body. Failure to protect the knee joint in daily life can easily lead to knee injury and discomfort symptoms such as knee swelling and pain [1, 2]. Knee osteoarthritis (KOA) is knee joint disease arising from the degeneration of knee joint and presents discomfort symptoms such as swelling, pain, snapping, and effusion [3]. Generally, the middle-aged and elderly people are high-risk people, and they are often accompanied by joint swelling and pain, joint effusion, limited activities, and other complications. The occurrence of this disease is related to overweight, age factors, excessive injuries, genetic factors, and other reasons [4–6]. There are many treatments for KOA, and different treatments can be adopted according to different causes. For example, in the early stage of the disease, drugs for removing dampness and blood stasis and promoting blood circulation are used for control, while acupuncture and massage are used for conservative treatment. When the symptoms are more serious, it is necessary to go to the hospital for examination and specific treatment after identifying the cause [7]. Because the knee bone joint is difficult to cure, special care is required in the later stage. Otherwise, it will recur [8]. Generally speaking, the early treatment of diseases will be very effective, which is also true for KOA.

There are many methods for clinical examination of knee joints, including X-ray plain film and CT. The X-ray can show whether the cartilage layer of the diseased joint becomes thinner or destroyed and whether the joint space becomes narrower, but other structures such as meniscus and ligament cannot be judged, and its clinical application value is limited [9, 10]. CT can find the degeneration of articular cartilage, the narrowing of joint space, the hyperosteogeny, and calcification, which is helpful to diagnose arthritis, but it can only see the changes in bone structure, and its diagnosis of arthritis caused by soft tissue is poor [11–13]. As a noninvasive examination technology, magnetic resonance imaging (MRI) does not have the radiation problem of X-ray or CT and can be repeated several times in a short period. Articular cartilage, meniscus, and ligament can be observed in various MRI sequences, assisting doctors in making more accurate assessment, which has become the most valuable method to evaluate knee cartilage, with the advantages of the high resolution of soft tissue, multiple parameters, and small diagnostic error [14]. Deep learning is a branch of machine learning, which attempts to use multiple processing layers with complex structures or multiple nonlinear transformations to abstract data at a high level [15]. It establishes neural networks that can simulate the human brain for analytical learning. It stimulates the mechanism of human brain to interpret data, such as images, texts, and sounds, and is also widely used in the field of clinical medical images [16].

To sum up, the combination of deep learning technology and medical images is a hot topic of research at present and has a broad development prospect. 104 KOA patients received the MRI scans with different sequences, and an image superresolution algorithm based on the improved multiscale wide residual network model was proposed for the image processing of MRI. The diagnostic accuracy of MRI images with different sequences for different injury grades was calculated to comprehensively evaluate the adoption value of the deep learning model combined with MRI images in the examination of KOA. It was hoped to provide help for the selection of imaging diagnosis of KOA.

## 2. Materials and Methods

### 2.1. Research Subjects

A total of 104 patients with KOA who were admitted to the hospital between October 20, 2018, and February 20, 2021, were recruited as the research subjects. All patients lived a normal life and had no history of high-intensity exercise training. This study had been approved by ethics committee of hospital. Patients and their families were aware of this study and had signed informed consent.

The inclusion criteria are as follows: (1) no past or recent history of major knee trauma, (2) no previous history of infectious diseases, (3) no previous surgical history, (4) no previous use of drugs affecting cartilage, (5) patients with complete clinical data, and (6) no contraindications for MRI examination.

The exclusion criteria are as follows: (1) poor MRI image quality, (2) patients without arthroscopic examination information, (3) patients with congenital or acquired knee deformity, and (4) body mass index (BMI) is too high or too low.

### 2.2. MRI Examination

3.0 T superconducting magnetic resonance imaging system was used, with 15 channel phased array surface coil. Before MRI scan, the patient was instructed to sit quietly for about 10 minutes and remove all metal objects on the body. Especially, whether cardiac pacemaker and coronary artery stent were installed should be figured out. The patient was in a supine position during scanning.

Conventional MRI scan, sagittal T1-weighted imaging (T1WI), proton density-weighted inhibition (PDWI-fs), coronal PDWI-fs, and axial T2-weighted imaging (T2WI) were performed first. Then, sagittal double-echo stable water excitation (3D-Dess-WE), T2 mapping, T2∗ mapping, and Tl mapping were carried out. The specific parameters are shown in Table 1.

In image processing, the multimodal MRI images were sent to a workstation for processing. Two experienced MRI diagnostic specialists assessed the severity of cartilage injury according to the Recht grading criteria and divided the cartilage into medial femur cartilage, lateral condyle cartilage, patellar cartilage, medial tibia cartilage, and femur trochlear cartilage. The relaxation time was also measured.

The sensitivity, specificity, and accuracy are calculated as follows.

(1) $$\begin{array}{c} \text{Specificity}=\frac{A_{4}}{A_{3}+A_{4}},\\ \text{Specificity}=\frac{A_{4}}{A_{3}+A_{4}},\\ \text{Accuracy rate}=\frac{A_{1}+A_{4}}{A_{1}+A_{2}+A_{3}+A_{4}}, \end{array}$$

where *A*_1_ indicates positive arthroscopy and positive MRI, *A*_2_ indicates positive arthroscopy and negative MRI, *A*_3_ indicates negative arthroscopy and positive MRI, and *A*_4_ indicates negative arthroscopy and negative MRI.

### 2.3. Image Superresolution Algorithm Based on Improved MSRN Model

Superresolution [17] refers to the reconstruction of corresponding high-resolution images from low-resolution images, which has important application value in monitoring equipment, satellite images, and medical images. MSRN [18] is a deep learning network model based on image superresolution, and its structure is shown in Figure 1.

In this structure, local residual learning can reduce computational complexity and improve network performance. Multiscale feature fusion can extract image features in different proportions and enable shared feature information of different branches. The operation can be expressed as follows.

(2) $$\begin{array}{c} F_{1}=\lambda \left(\alpha_{3*3}^{1}*H_{m-1}+c^{1}\right),\\ G_{1}=\lambda \left(\alpha_{5*5}^{1}H_{m-1}+c^{1}\right),\\ F_{2}=\lambda \left(\alpha_{3*3}^{2}*\left\lfloor F_{1},G_{1}\right\rfloor +c^{2}\right),\\ G_{2}=\lambda \left(\alpha_{5*5}^{2}*\left\lfloor G_{1},F_{1}\right\rfloor +c^{2}\right),\\ F^{\prime }=\alpha_{1*1}^{3}*\left\lfloor F_{2},G_{2}\right\rfloor +c^{2}, \end{array}$$

where *α* is the weight; *c* is the deviation; superscripts 1, 2, and 3 represent the layer where it is located at; 1∗1, 3∗3, and 5∗5 are the size of convolutional kernel; *λ*() is the RELU function; ⌊*F*_1_, *G*_1_⌋, ⌊*G*_1_, *F*_1_⌋, and ⌊*F*_2_, *G*_2_⌋ represent series operations; and *H* represents the number of network feature graphs.

The above network model only uses one scale convolution kernel to extract image features when obtaining high-frequency information from low-resolution images, which will greatly miss a lot of details of images. Therefore, on the basis of the above model, this study adds three branch networks of different scales, as shown in Figure 2.

The above model can convert RGB images into Ycbcr images and carry out superresolution reconstruction of Y channels. Suppose that a MR image has K channels; the model can be expressed as follows.

(3) δ⌢=argminδ∑i=1LR∗FδImiLRI,ImiHRIL,δ=α1,α2,⋯αn,c1,c2,⋯cn,

where Im^LRI^ is the low-resolution feature image, Im^HRI^ is the high-resolution feature image, *δ* represents the weight and deviation of the network, *L* denotes the number of images input, and *ℜ*∗ is the loss function to minimize the difference between the low-resolution feature image and the high-resolution feature image.

The network structure of the model is mainly composed of multiscale feature extraction block, wide residual block, and multiscale reconstruction. The multiscale feature extraction module can be expressed as follows.

(4) UMF=CONMF,×3ImLRI,

where CON_*MF*,×3_ represents feature extraction using the branch network of ×3.

The wide residual module needs to carry out wide residual feature extraction, feature fusion, local residual learning, and global residual learning. The wide residual feature extraction can be expressed as follows.

(5) $$\begin{array}{c} F_{1}=Z_{gn}\left(a_{3*3}^{1}*H_{m-1}+c^{1}\right),\\ G_{1}=Z_{gn}\left(a_{5*5}^{1}*H_{m-1}+c^{1}\right),\\ F_{2}=\lambda \left(a_{3*3}^{2}*\left\lfloor F_{1},{\text{G}}_{1}\right\rfloor +c^{2}\right),\\ G_{2}=\lambda \left(\alpha_{5*5}^{2}*\left\lfloor G_{1},F_{1}\right\rfloor +c^{2}\right). \end{array}$$

*Z*_*gn*_ indicates that the group normalization layer is used to normalize the feature graph, and the meanings of other letters are the same as before. Then, the fusion operation can be expressed as follows.

(6) $$\begin{array}{c} F^{\prime }=\alpha_{1*1}^{3}*\left\lfloor F_{2},G_{2}\right\rfloor +c^{2}. \end{array}$$

Local residual learning can improve the transmission of feature information and gradient flow in the network and obtain more detailed information, which can be expressed as follows.

(7) $$\begin{array}{c} H_{m}=F^{\prime }+H_{m-1}, \end{array}$$

where *H*_*m*_ represents local residual learning, and global residual learning can solve the problem of gradient disappearance in the training process of the network, which can be expressed as follows.

(8) $$\begin{array}{c} U_{GR}=U_{MF}+H_{M}, \end{array}$$

where *U*_*GR*_ represents global residual learning. Finally, multiscale reconstruction is carried out, and the final image can be expressed as follows.

(9) $$\begin{array}{c} {IM}_{re}=U_{3*3}\left(v_{\text{ups},\times 3}\left(U_{GR}\right)\right), \end{array}$$

where *IM*_*re*_ represents the obtained superresolution reconstructed image.

### 2.4. Evaluation of the Performance of Algorithm

The single-shot multibox detector (SSD) algorithm [19], superresolution convolutional neural network (SRCNN) algorithm [20], and enhanced deep superresolution (EDSR) algorithm are introduced [21] to compare with the improved widened MSRN structure model proposed in this study.

Peak signal noise ratio (PSNR) and structural similarity (SSIM) are used to evaluate for image reconstruction effects.

### 2.5. Statistical Methods

SPSS19.0 was used for data processing in this study. Mean ± standard deviation ($\bar{x}\pm s$) was used for measurement data, and percentage (%) was used for counting data. Pairwise comparison was performed by one-way ANOVA. The difference was statistically significant at *P* < 0.05.

## 3. Results

### 3.1. Performance Analysis of Improved Multiscale Wide Residual Network Structural Model

Firstly, the reconstructed image was subject to subjective evaluation (Figure 3). Compared with the original image, the reconstructed image by the four algorithms had significantly improved in terms of clarity and noise. The reconstructed image by the proposed model was clear enough with minimum noise and artifacts, and the overall quality was better than that processed by other algorithms.

Further quantitative index analysis (Figure 4) showed that the PSNR and SSIM of the reconstructed image by SRCNN algorithm were 30.41 dB and 0.892, respectively; for SSD, they were 26.11 dB and 0.749 dB, respectively; for EDSR algorithm, they were 27.84 dB and 0.788 dB, respectively; and for the model proposed in the study, they were 38.87 dB and 0.956, respectively. Evidently, PSNR and SSIM of reconstructed images by the model in this study were significantly higher than those of SRCNN, SSD, and EDSR algorithms, and the differences were statistically significant (*P* < 0.05).

### 3.2. Basic Information of the Subjects

As shown in Figure 5, in terms of gender, male patients (69 cases) were more than female patients (35 cases). In terms of age, most patients were 30-45 years old (67 cases), followed by <30 years old (27 cases) and >45 years old (10 cases). In terms of BMI, 18.5-23.9 kg/m^2^ patients were the most (63 cases), followed by >23.9 kg/m^2^ patients (21 cases) and <18.5 kg/m^2^ patients (20 cases). In terms of the affected knee joint, right knee was affected in 58 cases, and left knee was affected in 46 cases.

### 3.3. Imaging Data

Figure 6 shows the MRI data of a 28-year-old male. MRI image showed thickening of synovial membrane of the knee joint and multiple nodular and lobulated mixed signal shadows around the joint, most of which were long T1 and long T2 signal shadows. Multiple pomegranate seed-like low signal shadows were found inside, and serrated damage changes were observed in the lower femur and upper tibia subchondral segments.

Figure 7 shows the MRI data of a 45-year-old male. MRI images showed synovial thickening and joint cavity effusion. The thickened synovium presented low T1 and equal T2 signal shadows, and the boundary with adjacent tendons, ligaments, and muscles was not clear. Localized or extensive soft tissue swelling was observed around the knee, and T2WI presented high signals.

### 3.4. Arthroscopy Results

A total of 624 subareas of articular cartilage were found in 104 knee joints, and 295 cartilage lesions were detected by arthroscopy (Figure 8(a)), including 74 grade I lesions, 83 grade II lesions, 74 grade III lesions, and 64 grade IV lesions. Grade I lesions (Figure 8(b)) included 13 internal femoral condyles, 6 external femoral condyles, 10 internal tibial condyles, 4 external tibial condyles, 26 patella, and 15 femoral trochlea. Grade II lesions (Figure 8(c)) included 13 internal femoral condyles, 4 external femoral condyles, 11 internal tibial condyles, 5 external tibial condyles, 28 patella, and 22 femoral trochleae. Grade III lesions (Figure 8(d)) included 16 internal femoral condyles, 5 external femoral condyles, 14 internal tibial condyles, 6 external tibial condyles, 19 patella, and 14 femoral trochleae. Grade IV lesions (Figure 8(e)) included 14 internal femoral condyles, 4 external femoral condyles, 13 internal tibial condyles, 5 external tibial condyles, 17 patella, and 11 femoral trochleae.

### 3.5. Examination Results of Different MRI Sequences

With arthroscopy results as the gold standard, the diagnostic accuracy of PDWI-FS sequence for different injury grades was obtained (Figure 9). It was noted that the diagnostic accuracy of PDWI-FS sequence was 56.73% for grade I lesions, 60.42% for grade II lesions, 82.15% for grade III lesions, and 90.44% for grade IV lesions. The diagnostic accuracy of PDWI-FS sequence for grade III and IV lesions was significantly higher than that for grade I and II lesions, and the difference was significant (*P* < 0.05).

According to the consistency test, the Kappa consistency test value between PDWI-FS sequence and arthroscopy results was 0.517, indicating a moderate consistency.

With arthroscopy results as the gold standard, the diagnostic accuracy of 3D-DESS-WE sequence for different injury grades was obtained (Figure 10). The diagnostic accuracy of 3D-DESS-WE sequence was 84.72% for grade I lesions, 72.14% for grade II lesions, 85.15% for grade III lesions, and 96.74% for grade IV lesions. The diagnostic accuracy of 3D-DESS-WE sequence was high for all levels of lesions, especially for grade IV lesions, which reached more than 95%.

According to the consistency test, the Kappa consistency test value of 3D-DESS-WE sequence and the results of arthroscopy was 0.748, showing a strong consistency.

With arthroscopy results as the gold standard, the diagnostic accuracy of Tl mapping sequence for different injury grades was obtained (Figure 11). The diagnostic accuracy of Tl mapping sequence was 31.18% for grade I lesions, 40.68% for grade II lesions, 58.97% for grade III lesions, and 85.18% for grade IV lesions. The diagnostic accuracy of Tl mapping sequence in grade IV lesions was significantly higher than that in grade I lesions, grade II lesions, and grade III lesions (*P* < 0.05).

According to the consistency test, the Kappa consistency test value of Tl mapping sequence and arthroscopy results was 0.396, indicating a general consistency.

With arthroscopy results as the gold standard, the diagnostic accuracy of T2 mapping sequence for different injury grades was obtained (Figure 12). It was noted that the diagnostic accuracy of T2 mapping sequence was 60.55% for grade I lesions, 57.49% for grade II lesions, 68.06% for grade III lesions, and 92.31% for grade IV lesions. The diagnostic accuracy of T2 mapping sequence for grade IV lesions was significantly higher than that for grade I, II, and III lesions, and the difference was significant (*P* < 0.05).

According to the consistency test, the Kappa consistency test value of T2 mapping sequence and arthroscopy results was 0.578, indicating a moderate consistency.

With arthroscopy results as the gold standard, the diagnostic accuracy of T2∗ mapping sequence for different injury grades was obtained (Figure 13). It was noted that the diagnostic accuracy of T2∗ mapping sequence was 67.38% for grade I lesions, 70.13% for grade II lesions, 75.88% for grade III lesions, and 96.12% for grade IV lesions. The diagnostic accuracy of T2∗ mapping sequence for grade IV lesions was significantly higher than that for grade I lesions, grade II lesions, and grade III lesions, with significant difference (*P* < 0.05).

According to the consistency test, the Kappa consistency test value of T2∗ mapping sequence and arthroscopy results was 0.682, showing a strong consistency.

## 4. Discussion

Osteoarthritis, one of the common chronic diseases in the elderly, often causes patients with synovial joint injury and articular dysfunction [22]. As early osteoarthritis has no obvious symptoms, it can only be detected by functional imaging. Currently, X-ray, CT, and MRI are commonly used for knee examination [23]. In this study, KOA patients were examined by MRI. To improve image quality, an image superresolution algorithm based on an improved multiscale wide residual network model was proposed. Firstly, the superresolution reconstruction effect of the algorithm was analyzed. From the subjective evaluation, the image reconstructed by the model in this study was clear enough, with minimum noise and artifacts, and the overall quality was better than that processed by other algorithms. By further comparing the quantitative indicators of reconstructed images, it was noted that the PSNR and SSIM of the image reconstructed by the model in this study were significantly higher than those of SRCNN, SSD, and EDSR algorithms, and the differences were statistically significant (*P* < 0.05), in line with the research results of Vitaloni et al. [24]. Both PSNR and SSIM are conventional indicators used to evaluate image quality in academic field. The quantitative evaluation results being consistent with the above subjective evaluation results indicated that the superresolution reconstruction model has practical feasibility in MRI image processing and has clinical promotion value.

In this study, 104 KOA patients were recruited and underwent MRI scans. First, the basic data of patients were analyzed, and it was found that in terms of gender, male patients (69 cases) were more than female patients (35 cases); in terms of age, most patients were 30-45 years old (67 cases), followed by <30 years old (27 cases) and >45 years old (10 cases); in terms of BMI, 18.5-23.9 kg/m^2^ patients were the most (63 cases), followed by >23.9 kg/m^2^ patients (21 cases) and <18.5 kg/m^2^ patients (20 cases); and in terms of the affected knee joint, right knee was affected in 58 cases, and left knee was affected in 46 cases. Then, arthroscopic analysis found that grade I and grade II lesions concentrated on patella (26) and femoral trochlear (15), which was similar to the conclusions of previous studies that the patellar cartilage and the medial region of the femoral condyle were most vulnerable to cartilage injury [25]. In addition to involving the patella and femoral trochlea, grade III and grade IV lesions gradually developed into the medial and lateral articular cartilage. Next, with arthroscopic results as the gold standard, the diagnostic performance of MRI sequences was analyzed. The 3D-DS-WE sequence was found to be the best sequence for diagnosing KOA injury, with a high diagnostic accuracy of over 95% in grade IV lesions. The consistency test showed that the 3D-DESS-WE sequence and T2∗ mapping sequence had a strong consistency with the results of arthroscopy, and the Kappa consistency test values were 0.748 and 0.682, respectively. The results showed that 3D-DS-WE sequence and T2∗ mapping sequence were acceptable in the diagnosis of KOA injury and superior to other sequences.

## 5. Conclusion

104 KOA patients received MRI scans with different sequences. Then, an image superresolution algorithm based on the improved multiscale wide residual network model was proposed for the image processing of MRI. The consistency test showed that the 3D-DESS-WE sequence and T2∗ mapping sequence had a strong consistency with the results of arthroscopy, and the Kappa consistency test values were 0.748 and 0.682, respectively. However, the cases are selected from a single source with regional limitations, and whether combined detection of different sequences will improve the diagnostic performance of KOA injury is not further discussed. The follow-up research should focus on this problem to strengthen the findings of the study. All in all, this study provides a reference for the combined application of deep learning model and image technology in the diagnosis of KOA.

## Figures and Tables

**Figure 1:** Multiscale residual network structure.

**Figure 2:** Improved widened multiscale residual network structure model.

**Figure 3:** Reconstruction results of MRI images by different algorithms. (a)–(e) are the original image, reconstructed image by SRCNN algorithm, reconstructed image by SSD algorithm, reconstructed image by EDSR algorithm, and reconstructed image by the model in the study.

**Figure 4:** Comparison of PSNR and SSIM of reconstructed images by four algorithms. # represents significant difference between algorithms (*P* < 0.05).

**Figure 5:** Basic information of subjects.

**Figure 6:** Male, 28 years old, presented with sudden redness and pain of the right knee joint for 3 days. (a) and (b) are sagittal T2WI, while (c) and (d) are transverse T2WI.

**Figure 7:** Male, 45 years old, chief complaint: recurrent pain in the knuckles of both hands and toes for 5 years, recurring 1 week before. (a) and (b) are sagittal T2WI, while (c) and (d) are transverse T2WI.

**Figure 8:** Arthroscopy results. (a) The grade of cartilage injury. (b) The distribution of grade I lesions. (c) The distribution of grade II lesions. (d) The distribution of grade III lesions. (e) The distribution of subareas of grade IV lesions.

**Figure 9:** Diagnostic accuracy of PDWI-FS sequence for different injury grades. A and B indicate that pairwise comparison has statistical significance (*P* < 0.05).

**Figure 10:** Diagnostic accuracy of 3D-DESS-WE sequence for different injury grades. A and B indicate that pairwise comparison has no statistical significance (*P* < 0.05).

**Figure 11:** Diagnostic accuracy of Tl mapping sequence for different injury grades. A and B indicate that pairwise comparison has no statistical significance (*P* < 0.05).

**Figure 12:** Diagnostic accuracy of T2 mapping sequence for different injury grades. A and B indicate that pairwise comparison has no statistical significance (*P* < 0.05).

**Figure 13:** Diagnostic accuracy of T2∗ mapping sequence for different injury grades. A and B indicate that pairwise comparison has no statistical significance (*P* < 0.05).

**Table 1:** Sequence scanning parameters.

Parameter	3D-DESS-WE	T2 mapping	T2∗ mapping	Tl mapping
Time of echo (TE)	6 ms	15.6 ms	10.5 ms	2.55 ms
Time of repetition (TR)	13.55 ms	1500 ms	550 ms	25 ms
Band width	220 Hz	/	/	/
Vision	145 × 145 mm	145 × 145 mm	145 × 145 mm	145 × 145 mm
Resolution	265 × 265	350 × 350	315 × 315	350 × 350
Layer thickness	/	3.6 mm	3.6 mm	3.6 mm
Layer distance	/	0.8 mm	0.8 mm	0.8 mm

## Data Availability

The data used to support the findings of this study are available from the corresponding author upon request.
